# Transforming growth factor-β1-regulated Fas/FasL pathway activation suppresses nucleus pulposus cell apoptosis in an inflammatory environment

This article has been retracted.

**DOI:** 10.1042/BSR20191726

**Published:** 2020-02-04

**Authors:** Jingjing Xie, Bo Li, Bing Yao, Pingchao Zhang, Lixin Wang, Hua Lu, Xuan Song

**Affiliations:** Department of Orthopedic Surgery, Xinhua Hospital Affiliated to Shanghai Jiao Tong University School of Medicine, Chongming Branch, Shanghai 202150, China

**Keywords:** apoptosis, Fas/FasL, nucleus pulposus, TGF-β1, TNF-α

## Abstract

Background: During disc degeneration, inflammatory cytokine tumor necrosis factor (TNF)-α is correlated with nucleus pulposus (NP) cell apoptosis. Transforming growth factor (TGF)-β1 has the potential to regenerate degenerative disc.

Objective: To investigate the protective role of TGF-β1 against TNF-α-mediated NP cell apoptosis and the underlying mechanism.

Methods: Rat NP cells were treated with TNF-α (100 ng/ml) for 48 h. TGF-β1 was added into the culture medium to investigate its protective effects against TNF-α-induced NP cell apoptosis. Exogenous FasL was used to investigate the potential role of the Fas/FasL pathway in this process. Flow cytometry assay was used to analyze NP cell apoptosis. Real-time PCR and Western blotting were used to analyze gene and protein expression of apoptosis-related molecules.

Results: In TNF-α-treated NP cells, TGF-β1 significantly decreased NP cell apoptosis, declined caspase-3 and -8 activity, and decreased expression of Bax and caspase-3 (cleaved-caspase-3) but increased expression of Bcl-2. However, exogenous FasL partly reversed these effects of TGF-β1 in NP cells treated with TNF-α. Additionally, expression of Fas and FasL in TNF-α-treated NP cells partly decreased by TGF-β1, whereas exogenous FasL increased expression of Fas and FasL in NP cells treated with TGF-β1 and TNF-α.

Conclusion: TGF-β1 helps to inhibit TNF-α-induced NP cell apoptosis and the Fas/FasL pathway may be involved in this process. The present study suggests that TGF-β1 may be effective to retard inflammation-mediated disc degeneration.

## Introduction

Low back pain (LBP) is a common ailment that affects patient’s life quality and causes a heavy financial burden on the healthcare system [1]. Intervertebral disc degeneration (IDD) is regarded as a main contributor to LBP [2]. Although the traditional treatments including conservative therapy and disectomy are effectual to some degree, they mainly target symptom relief but not the pathogenesis of the problem. Hence, lot of researchers declare that the early prevention of degeneration and restoration of the disc’s biological function are the ideal approaches to biologically treat IDD.

During disc degeneration, progressive decline of proteoglycans and tissue dehydration are the major pathological characteristics of disc matrix, leading to destruction of disc structure and spine function [3]. Nucleus pulposus (NP), the central gelatinous-like structure, is rich in proteoglycans [4]. The proteoglycan with large amount of negative charges produces a hypermostic niche and thus a high hydration within the NP tissue, which is necessary for maintaining the normal mechanical function of the intervertebral disc (IVD) [5]. Currently, the pathophysiological mechanism for IDD is unclear, but it has been established that cell apoptosis participates in this pathological process [6]. Recent findings have showed that apoptosis-induced decrease in the number of NP cell directly leads to alternation of composition of the NP extracellular matrix (ECM) [7,8]. Therefore, the inhibition and/or attenuation of disc NP cell apoptosis may be a promising treatment that retards disc degeneration.

Tumor necrosis factor (TNF)-α, a member of the TNF superfamily of ligands, is highly expressed in the degenerative and herniated human IVD tissues compared with the non-degenerative IVD tissues [9]. Importantly, TNF-α is thought to be responsible for disc degeneration [10,11]. Currently, increasing evidence has supported the involvement of TNF-α in mediating NP cell apoptosis. For example, TNF-α significantly increases apoptosis rate and up-regulates the expressions of p53 and caspase 3 in NP cells from the human degenerative disc NP samples [12]. Similarly, rabbit NP cells undergo apoptosis and display apoptosis-associated morphological changes following exposure to TNF-α *in vitro* [13]. Thus, TNF-α plays an important role in promoting NP cell apoptosis during disc degeneration.

Transforming growth factor (TGF)-β1 is a polypeptide belonging to the TGF-β superfamily of cytokines. It has a wide range of regulatory functions on cellular growth, proliferation, differentiation and apoptosis [14]. A previous study has demonstrated that the expression of both TGF-β and its receptor were decreased in the degenerative disc cells [15]. Moreover, TGF-β-mediated signaling pathways plays an essential role in the growth and maintenance of disc tissues [16]. Additionally, TGF-β is able to antagonize inflammatory cytokine-induced up-regulation of matrix metalloproteinase 3 in disc NP cells [17,18] and inflammation-related pain in a rat model [19]. To further determine whether TGF-β1 has a protective effect against NP cell apoptosis, we mainly investigated the effects of TGF-β1 on the TNF-α-mediated NP cell apoptosis and the potential role of Fas/FasL pathway in the present study.

## Materials and methods

### NP cell isolation and culture

Lumbar discs (L2–L5) from 35 healthy Sprague–Dawley rats (aged 2 months, female or male, 460 ± 24 g in weight) were harvested immediately under the sterile conditions after they were killed by excessive carbon dioxide inhalation. Then, the central NP tissue was removed, and the inner annulus fibrosus (AF) and the transition zone (TZ) were separated under a dissecting microscope. The separated NP tissue was sequentially digested with 0.25% type II collagenase for 10 min and 0.2% trypsin with EDTA (1 mmol/l) for 5 min, as previously described [20]. Thereafter, NP cell pellets were transferred to DMEM/F12 medium (HyClone, U.S.A.) supplemented with 20% FBS (Gibco, U.S.A.) and cultured in a humidified atmosphere (20% O_2_, 5% CO_2_ at 37°C). When NP cells grew to 70–80% confluence, they were dissociated using 0.25% trypsin (HyClone, U.S.A.) and further subcultured. Second-passage NP cells (Figure 1) in monolayer culture were used for the following experiments.

**Figure 1:** Flow cytometry analysis of NP cell apoptosis (**A**) Representative images of flow cytometry analysis. (**B**) Histogram of apoptosis rate in different groups. Data are expressed as mean ± SD, *n*=3. *: Indicates a significant difference (*P*<0.05) between two groups.

### Experimental groups

To study the role of TGF-β1 on TNF-α-mediated NP cell apoptosis and the potential mechanism, four groups were designed in the present study. Group I: NP cells were free from exogenous intervention. Group II: NP cells were treated with TNF-α (100 ng/ml [13], R&D Systems, U.S.A.). Group III: NP cells were treated with TNF-α (100 ng/ml) and TGF-β1 (10 ng/ml [21], R&D Systems, U.S.A.). Group IV: NP cells were treated with TNF-α (100 ng/ml), TGF-β1 (10 ng/ml) and FasL (20 ng/ml [22], R&D Systems, U.S.A.). Group V: NP cells were treated with TNF-α (100 ng/ml), TGF-β1 (10 ng/ml), FasL (20 ng/ml) and ZB4 (500 ng/ml, Millipore, Billerica, MA, U.S.A.). After 48 h, NP cells in each group were collected and used to analyze cellular apoptosis and expression of Fas and FasL. Because several previous studies have verified that a concentration of 100 ng/ml TNF-α could induce disc NP cell apoptosis, the concentration of TNF-α used in the present study was 100 ng/ml [23,24].

### Cell apoptosis analysis

Cell apoptosis was assessed using annexin V-FITC/PI staining method (Beyotime, China) according to the manufacturer’s instructions. Briefly, after NP cells were incubated with different test compounds for 48 h, they were washed with cold phosphate buffer solution (PBS) and then resuspended in binding buffer. Then, NP cells were stained with 5 μl Annexin V-FITC and 10 μl PI for 10 min at room temperature. Finally, the stained NP cells were subjected to a flow cytometry machine (Japan PHENIX Company) to analyze cell apoptosis. NP cells that were positively stained with Annexin V-FITC and negatively stained with PI, or both positively stained were considered as apoptotic cells.

### Capase-3 and 8 activity measurement

Caspase-3 and -8 activity was evaluated using the caspase-3/-8 activity detection kits (Beyotime, China). Briefly, after NP cells were incubated with different test compounds for 48 h, the protein supernatant was extracted using the lysis solution. Then, their activities were measured according to the manufacturer’s instructions. Finally, the optical density (OD) at a wavelength of 405 nm was measured to calculate the activity of caspase-3 and -8 which was normalized to the total protein.

### Real-time PCR analysis

After NP cells were incubated with different test compounds for 48 h, total RNA was extracted with TRIzol reagent (Invitrogen, U.S.A.) based on the manufacturer’s directions. The single-stranded cDNA was prepared from 1 μg of total RNA using a reverse transcription kit (Roche). Specific cDNA templates were then amplified by PCR using the specific primers (Table 1, Sangon, Biotech Co., Ltd., China). PCR amplification reaction was performed in a final system of 25 μl containing primers, cDNA samples and SYBR Green qPCR Mix (Dongsheng Biotech, China). The cycling parameters were: 5 min at 95°C, followed by 40 amplification cycles of 30 s at 95°C, 30 s at 56°C and 30 s at 72°C. *β-actin* was used as a reference gene and the relative gene expression was calculated by the method of 2^―ΔΔ*C*_t_^.

**Table 1:** Primers of target genes

Gene	Forward (5′–3′)	Reverse (5′–3′)
*β-actin*	CCGCGAGTACAACCTTCTTG	TGACCCATACCCACCATCAC
*Bcl-2*	GGGGCTACGAGTGGGATACT	GACGGTAGCGACGAGAGAAG
*Bax*	GGCGAATTGGCGATGAACTG	CCCAGTTGAAGTTGCCGTCT
*Caspase 3*	GGAGCTTGGAACGCGAAGAA	ACACAAGCCCATTTCAGGGT

### Western blotting assay

The expression of cleaved caspase-3, Bcl-2, Bax, Fas and FasL was analyzed by Western blotting. β-actin was used as the internal control. Briefly, after total protein was extracted from NP cells with RIPA buffer (Beyotime, China), protein concentration was determined by the BCA assay kit (Beyotime, China). Then, equal protein samples in each group were sequentially subjected to SDS-PAGE and transferred to the PVDF membrane. After the PVDF membranes were blocked with 5% bovine serum albumin (BSA) for 1 h at 37°C, they were incubated overnight at 4°C with corresponding primary antibodies (cleaved caspase-3: Cell Signaling Technology, #9661; Bcl-2: Proteintech, 12789-1-AP; Bax: Proteintech, 50599-2-Ig; Fas: Santa Cruz Biotechnology, sc-1023; FasL: Santa Cruz Biotechnology, sc-19681; β-actin: Santa Cruz Biotechnology, sc-130065), followed by incubation with horseradish peroxidase–conjugated secondary antibodies (Cell Signaling Technology, 1:1000) for 1 h at room temperature. Finally, PVDF membranes were treated with ECL Plus (Amersham Pharmacia Biotech, Umea, Sweden). Gray value of protein bands was analyzed using the ImageJ software (National Institutes of Health, U.S.A.). Expression of all target proteins was normalized to expression of β-actin.

### Statistical analysis

All data in the present study were expressed as mean ± SD. All experiments were performed in triplicate to ensure consistency. SPSS 11.0 software (Chicago, IL, U.S.A.) was used for the statistics. When the homogeneity test for variance was completed, data were compared using one-way analysis of variance (ANOVA), and the post hoc test was determined by the LSD test. The *P*-value of 0.05 or less was considered a significant difference.

## Results

### TGF-β1 partly attenuated TNF-α-induced NP cell apoptosis

Results showed that NP cell apoptosis in the TNF-α group was significantly increased compared with the control group, and TGF-β1 partly attenuated NP cell apoptosis in the TNF-α group. However, addition of exogenous FasL partly attenuated the protective role of TGF-β1 in the TNF-α group (Figure 1).

### TGF-β1 partly decreased caspase-3/8 activity of TNF-α-treated NP cells

Results showed that activity of both caspase-3 and caspase-8 in the TNF-α group were significantly increased compared with the control group, and TGF-β1 partly decreased their activities in the TNF-α group. Oppositely, their activities in the TNF-α+TGF-β1 group were partly increased again by the addition of exogenous FasL (Figure 2).

**Figure 2:** Caspase-3 and caspase-8 activity measurement of NP cells Data are expressed as mean ± SD, *n*=3. *: Indicates a significant difference (*P*<0.05) between two groups.

### TGF-β1 partly reversed gene ecpression profile of apoptosis-related molecules in TNF-α-treated NP cells

TNF-α significantly down-regulated gene expression of anti-apoptotic molecules (Bcl-2) compared with the control group, whereas TGF-β1 partly increased Bcl-2 mRNA expression in the TNF-α group. However, exogenous FasL decreased Bcl-2 mRNA expression in the TNF-α+TGF-β1 group. In addition, gene expression of caspase-3 and Bax showed an opposite trend among these groups (Figure 3).

**Figure 3:** Gene expression of apoptosis-related molecules (Bcl-2, Bax and caspase-3) of NP cells Data are expressed as mean ± SD, *n*=3. *: Indicates a significant difference (*P*<0.05) between two groups.

### TGF-β1 partly reversed protein expression profile of apoptosis-related molecules in TNF-α-treated NP cells

Results showed that TNF-α significantly increased protein expression of cleaved-caspase-3 and Bax compared with the control group, and addition of TGF-β1 partly decreased their expressions. Importantly, exogenous FasL in the TNF-α+TGF-β1 group partly increased their protein expressions. Inversely, protein expression of Bcl-2 showed an opposite pattern compared with cleaved caspase-3 and Bax among these groups (Figure 4).

**Figure 4:** Protein expression of apoptosis-related molecules (Bcl-2, Bax and caspase-3) of NP cells Data are expressed as mean ± SD, *n*=3. *: Indicates a significant difference (*P*<0.05) between two groups.

### TGF-β1 partly decreased protein expression of Fas/FasL in TNF-α-treated NP cells

To evaluate the potential role of the Fas/FasL pathway, we analyzed protein expression of Fas and FasL. Results showed that TNF-α simultaneously increased their protein expressions compared with the control group, but their expressions of TNF-α-treated NP cells decreased by addition of TGF-β1. However, exogenous FasL partly increased protein expressions of both Fas and FasL of NP cells in the TNF-α+TGF-β1 group (Figure 5).

**Figure 5:** Protein expression of Fas and FasL of NP cells Data are expressed as mean ± SD, *n*=3. *: Indicates a significant difference (*P*<0.05) between two groups.

## Discussion

Disc degeneration is a common degenerative disease in adults. Until now, the accurate pathogenesis of disc degeneration is not clear. It has been established that NP cell apoptosis is the main cause of disc degeneration and gradually increases with advancing age [6,25,26]. Besides, increased content of inflammatory cytokines is another important feature within the degenerative disc NP region [27]. In the present study, we confirmed that inflammatory cytokine TNF-α promoted NP cell apoptosis and found that TGF-β1 was potentially helpful to attenuate TNF-α-mediated NP cell apoptosis through regulating the Fas/FasL pathway. The present study provides that TGF-β1 may be a promising growth factor to attenuate inflammation reaction-induced NP cell apoptosis during disc degeneration.

Apoptosis is commonly termed as Type I programmed cell death, which is a cell self-destruction process involved in lots of biological events, such as tissue development, tissue homeostasis and the removal of needless cells. During disc degeneration, some detrimental pathological factors induce uncontrolled or overmany apoptosis, which can lead to the decrease in ECM content through significant loss of IVD cells. It is well known that inflammation plays a critical role in the pathology of IDD. To investigate the accurate role of inflammation in mediating disc degenerative changes, many researchers carried out studies in this field. Specifically, several studies have demonstrated that interleukin-1β increases NP cell apoptosis ratio or sensitizes NP cell to certain pathological factors-mediated cellular apoptosis [20,28–34]. Similarly, there are evidence that TNF-α is also an inductive factor to cause unwanted NP cell apoptosis [24,35]. In line with this, we confirmed those previous studies that TNF-α significantly promoted NP cell apoptosis *in vitro*. For example, we found that TNF-α significantly increased NP cell apoptosis and caspase-3/-8 activity, up-regulated expression of Bax and caspase-3, and down-regulated expression of Bcl-2 in the present study. Collectively, these results indicate that inhibition of inflammation-induced NP cell apoptosis may be a promising approach to alleviate disc degeneration.

Fas/FasL system is a well-characterized cellular apoptosis pathway [36]. Fas protein expresses in a wide variety of cell types, but FasL protein expresses in a restricted range of cell types. FasL often acts as a cell death-triggering ligand to induce apoptosis upon binding to the Fas protein [36,37]. Previously, different roles of FasL have been suggested in regulating disc cell biology. Some reports have indicated that FasL plays an important role in the development and the immune privilege of discs [38,39]. On the other hand, FasL was found to be closely related with disc cell apoptosis [40] and thought to be responsible for disc degeneration [39]. In this study, we found that TNF-α significantly increased Fas and FasL protein expression. In light of the aggravated NP cell apoptosis in the TNF-α-treated NP cells, and the positive role of Fas/FasL in mediating cellular apoptosis, we deduce that TNF-α may cause NP cell apoptosis through activating the Fas/FasL pathway.

TGF-β is a cytokine that participates in various cellular processes. It can bind to the transmembrane serine/threonine protein kinase receptors and then activate many downstream pathways, such as TGF/Smad pathway and RhoA/ROCK pathway [14,41,42]. Previously, several studies have reported the positive effects of TGF-β family on disc cells. Risbud et al. [43] demonstrated that TGF-β3, an isoform of the TGF-β family, maintained NP cell viability and enhanced phenotypic matrix deposition. Hu et al. [21] demonstrated that TGF-β3 induced chondroitin polymerizing factor (ChPF) expression through activating the Smad3 and ultimately promoted biosynthesis of sulfated glycosaminoglycan (sGAG) in NP cells. Yang et al. [44] showed that transplantation of mescenchymal stem cells combined with pure fibrinous gelatin and TGF-β1 exhibited a slower decrease in disc height index and a higher collagen II content. In this study, we found that TGF-β1 inhibited TNF-α-mediated NP cell apoptosis, and that the protein expression of Fas/FasL was decreased by the addition of TGF-β1. These results are consistent with previously reported protective effects of TGF-β against disc degeneration. However, an *in vivo* study is needed to further verify its positive effects against TNF-α-mediated NP cell apoptosis.

Several important issues need to be discussed here. In the present study, the NP cells were isolated from the rat disc NP tissue. Rat disc NP tissue is proved to contain lots of notochordal cells which differ from disc NP cells in some aspects. Moreover, there are no specific cellular markers to accurately distinguish NP cells from notochordal cells currently [45]. Therefore, the isolated disc NP cells may not be pure NP cells in the present study. The existence of notochordal cells may bring some interference to our results. In addition, we did not use the specific inhibitors (i.e. the Fas inhibitor ZB4) or silence some factors in the Fas/FasL pathway to exemplify the molecular link between TGF-β1 and apoptosis via the Fas/FasL pathway. The present study is just a preliminary research of our team. In the future, we will further study it if possible.

## Conclusion

In conclusion, we investigated the protective role of TGF-β1 against TNF-α-mediated NP cell apoptosis, and the potential role of the Fas/FasL pathway in this process in the present study. Our results confirmed that TNF-α could cause NP cell apoptosis and revealed that TGF-β1 is effective to attenuate TNF-α-mediated NP cell apoptosis through regulating the Fas/FasL pathway. The present study is helpful to shed a deeper understanding toward disc degeneration.

## Abbreviations

Bax: bcl-2 associated X protein
Bcl-2: b-cell lymphoma-2
ECM: extracellular matrix
IDD: intervertebral disc degeneration
IVD: intervertebral disc
LBP: low back pain
NP: nucleus pulposus
PI: propidium iodide
TGF: transforming growth factor
TNF: tumor necrosis factor
